The article "Research on the Green Production Motivation of New Agricultural Business Entities: Benefit Perception and Environmental Regulation" was published in 2022. Journal: J Environ Public Health.

# Research on the Green Production Motivation of New Agricultural Business Entities: Benefit Perception and Environmental Regulation

**DOI:** 10.1155/2022/9182725

**Published:** 2022-07-30

**Authors:** Yufeng Li, Zihan Zhu, Pu Xu

**Affiliations:** School of Economics and Management, Shanghai Ocean University, 201306 Shanghai, China

## Abstract

The new agricultural business entities are key carriers of modern agriculture in China, and increasing their willingness to engage in green production is critical to the country's agricultural green transformation. The Economic and Social Man Hypothesis and Externality Theory are used to construct analysis models of the green production willingness of new agricultural business entities based on 106 survey data points from Shanghai to study the impact of benefit perception, environmental regulation, and their synergy on the green production willingness of new agricultural business entities. The results show that (1) benefit perception and environmental regulation can significantly improve the willingness of new agricultural business entities to engage in green production. Economic benefit perception, ecological benefit perception, guidance regulation, and restraint regulation are all important influencing factors. (2) There is a significant synergy between ecological benefit perception and environmental regulation in increasing the willingness of new agricultural business entities to engage in green production. Further research revealed that the synergistic item of ecological benefit perception and guidance regulation, as well as the synergistic item of ecological benefit perception and restraint regulation, significantly increases the willingness of new agricultural business entities to green production. The government should strengthen the perceptions of the economic and ecological benefit of new agricultural business entities to green production; change the incentive regulation and strengthen guidance regulation and restraint regulations; enhance the synergy between ecological benefit perception and guidance regulation; and enhance the synergy between ecological benefit perception and restraint regulation.

## 1. Introduction

Due to a heavy reliance on inputs such as chemical fertilizers and pesticides, China's agricultural total economic output has steadily increased since reform and opening [1]. However, widespread use of inputs such as fertilizers and pesticides has also led to increasing environmental degradation and resource scarcity [2]. This contradicts the United Nations' proposal for green development in 2002 and the concept of green development proposed at the Communist Party of China's 18th Central Committee's Fifth Plenary Session [3]. The extensive management methods of traditional agriculture in China are in urgent need of green innovation. To this end, relevant policies have been successively promulgated in recent years, from the Central Committee of the Communist Party of China to various ministries and commissions, emphasizing “adhering to the concept of agricultural green development” and “promoting agricultural green production methods.” ([4] The green transformation of China's agriculture has yielded preliminary results as a result of a series of policies, but its extensive management methods, which are based primarily on resource consumption, have not been fundamentally altered. The difficulty in changing China's extensive agricultural management methods, as well as the agricultural high carbon emissions and nonpoint source pollution [5, 6], is due to agricultural business entities' lack of willingness to switch to green production [7].

Traditional farmers and new agricultural business entities (including large grain growers, family farms, agricultural cooperatives, and leading enterprises) make up the majority of China's agricultural business entities. Traditional farmers are the microunit of agricultural production in China [2], but scholars have pointed out that they face a number of problems, including low risk tolerance, serious part-time jobs, smallholder economic awareness, and scattered and fragmented land, all of which impede their agricultural green production [8–10]. As a key cultivation subject in China's rural revitalization strategy, the overall number of new agricultural business entities has exploded in recent years. They not only avoid the aforementioned problems of limiting traditional farmers' green production, but they can also drive and control traditional farmers' green production [11, 12]. To summarize, increasing the willingness of new agricultural business entities to engage in green production is critical to promoting China's green transformation of agriculture, thereby realizing China's carbon peaking strategy and relieving environmental pressure.

## 2. Literature Review

As the core of civil production and an indispensable part of the national economy, agricultural industry plays a role in many aspects, but it also produces a large number of carbon emissions harmful to the environment [13, 14]. Agricultural green production is a method of production that not only increases agricultural production and profitability, but also reduces pollution and resource waste, with the goal of combining economic and ecological benefit [15]. The new agricultural business entities in China belong to “Economic and Social Man,” which are both self-interested and altruistic [16]. Their perceptions of economic and ecological benefit of agricultural green production are the primary internal motivators influencing their willingness to green produce [17]. Furthermore, agricultural green production is categorized as an “external economy.” However, China's market for “green agricultural products” is lagging, preventing new agricultural business entities from fully capitalizing on the positive externality of green agricultural production. The government can promote the development of agricultural green production by increasing the punishment for environmental damage and the reward for green production [18, 19]. Environmental regulation by the government has become an important external factor in the direction of agricultural green production [20–22]. Therefore, environmental regulation (guidance, incentive, and restraint) is the key external motivator influencing new agricultural business entities' willingness to engage in green production [23]. In conclusion, benefit perception and environmental regulation are important factors influencing the willingness of new agricultural business entities to produce green. Understanding how these two factors act is essential for increasing the willingness of new agricultural business entities to produce green products.

Academics have investigated the impact of benefit perception and environmental regulation on agricultural green production willingness. From the perspective of benefit perception, X H Zhao et al. discovered that traditional farmers' willingness to switch to green production is influenced by their perception of ecological benefit, but the study excluded economic benefit perception [24]; Y Z Huang et al. discovered that both economic and ecological benefit perceptions can encourage traditional farmers to switch to green production, but the impact mechanism of ecological benefit perception on traditional farmers' willingness to green production is difficult to explain due to the Cost-Benefit Theory's limitations [2]. From the perspective of environmental regulation, H L Zhang et al. and Y W Du et al. both found that guidance and incentive regulations can increase the willingness of traditional farmers to produce green products [23, 25]. In addition, D Liu and J Sun discovered that the combination of environmental regulation and market profit can motivate traditional farmers to produce green products. In an imperfect green market, environmental regulation can compensate for the lack of market profits [26].

This paper is based on the aforementioned research, and the potential marginal contributions are primarily reflected in the following: (1) the majority of current research on China's agricultural green production focuses on traditional farmers while ignoring the diversity of new agricultural business entities and their “leadership” role in promoting the green transformation of agriculture. The focus of this study will be on new agricultural business entities. (2) The majority of existing benefit perception research is based on traditional theories such as the Economic Man Hypothesis and the Social Man Hypothesis, which can only be investigated for the perception of economic or ecological benefit, but not both. This paper makes an attempt to improve by using the relatively new Economic and Social Man Hypothesis. (3) There is much existing literature on the willingness of agr1icultural green production based on benefit perception or environmental regulation. However, few scholars have studied the synergy between benefit perception and environmental regulation. This paper will attempt to conduct research from a synergistic perspective.

## 3. Theoretical Hypothesis

### 3.1. Benefit Perception and the Economic Social Man Hypothesis

According to the “Economic and Social Man Hypothesis,” a man has self-interest, altruism, and detriment. In socialist market economic activities with Chinese characteristics, the behavior of “economic and social man” is primarily guided and regulated by altruism and dominated by self-interest [16]. According to the Economic and Social Man Hypothesis, the fundamental internal motivations that affect the social and economic activities of China's new agricultural business entities are self-interest and altruism. The United Nations Environment Program defines agricultural “green production” as combining economic and ecological benefit. The Economic and Social Man Hypothesis is used in this paper to investigate the impact of benefit perception on the willingness of new agricultural business entities to engage in green production. It is as follows: motivated by self-interest, the perception of economic benefit has a positive impact on the willingness of new agricultural business entities to engage in green production. Motivated by altruism, the perception of ecological benefit has a positive impact on the willingness of new agricultural business entities to engage in green production. To summarize, the following hypotheses are proposed in this paper:

  H1a: the willingness of new agricultural business entities to produce green is positively influenced by their perception of economic benefit
  H1b: the willingness of new agricultural business entities to produce green is positively influenced by their perception of ecological benefit

### 3.2. Environmental Regulation and Externality Theory

According to the Externality Theory [27], externalities are classified as “external economy” or “external diseconomy.” “External economy” refers to the economic behavior that has a positive and beneficial impact on others and the environment, whereas “external diseconomy” refers to the opposite [28]. According to the Externality Theory, agricultural green production belongs to the “external economy.” However, China's current market for “green agricultural products” is imperfect, and fully capitalizing on its positive externalities is difficult. It is necessary to rely on government environmental regulation to promote green agricultural production [29]. Environmental regulation, which includes guidance regulation, incentive regulation, and restraint regulation, refers to the government's adoption of relevant regulatory policies to coordinate the ecological environment and economic development [30, 31]. Guidance regulation refers to the government's promotion of green agricultural production; incentive regulation refers to the government's subsidizing green production technology, green inputs, and rewarding agricultural green production; restraint regulation refers to the government promulgating a series of laws and regulations to restrict nongreen agricultural production. According to some studies, guidance regulation and incentive regulation are important in promoting traditional farmers' green production, but restraint regulation has little impact because traditional farmers are difficult to supervise and restrain [23, 32]. The new agricultural business entities, unlike traditional farmers, are large-scale operations, making it easier for the government to implement management and control regulations. As a result, this paper believes that environmental regulation and three regulatory tools (guidance, incentive, and restraint regulation) have a positive impact on new agricultural business entities' willingness to engage in green production. Based on the preceding analysis, this paper proposes hypotheses H2, H2a, H2b, and H2c:

  H2: environmental regulation increases the willingness of new agricultural business entities to engage in green production
  H2a: guidance regulation increases the willingness of new agricultural business entities to engage in green production
  H2b: incentive regulation increases the willingness of new agricultural business entities to engage in green production
  H2c: restraint regulation increases the willingness of new agricultural business entities to engage in green production

### 3.3. The Synergy of Benefit Perception and Environmental Regulation

Self-interest is human nature. Self-interest will drive new agricultural business entities to pursue the economic benefit of green production. However, China's market for “green agricultural products” is still developing, and the economic benefits of green production are not yet fully realized. Because the economic benefits of green production have yet to be realized, the government's use of environmental regulation to promote green production of new agricultural business entities rather than perfecting the “agricultural market” may cause resistance from new agricultural business entities to agricultural green production. As a result, this paper contends that the synergy between economic benefit perception and environmental regulation has a negative impact on new agricultural business entities' willingness to engage in green production. Altruism is human nature, and altruism will drive new agricultural business entities to pursue the ecological benefit of agricultural green production, which are obvious. The perception of ecological benefit will drive new agricultural business entities to obey environmental regulation promotion on the willingness of green production, and environmental regulation will amplify the positive impact of the perception of ecological benefit on the willingness of green production of new agricultural business entities. As a result, this paper contends that the synergy between ecological benefit perception and environmental regulation has a positive impact on new agricultural business entities' willingness to engage in green production. To summarize, hypotheses H3a and H3b are proposed:

  H3a: the synergy between economic benefit perception and environmental regulation has a negative impact on new agricultural business entities' willingness to engage in green production
  H3b: the synergy between ecological benefit perception and environmental regulation has a positive impact on new agricultural business entities' willingness to engage in green production

The synergy roadmap of benefit perception and environmental regulation is shown in Figure 1.

## 4. Materials and Methods

### 4.1. Data Collection

The research team distributed questionnaires on green production willingness to new agricultural business entities in nine major agricultural areas in Shanghai. First of all, the research team thoroughly explained the content, benefits, and drawbacks of agricultural green production to the new agricultural business entities under consideration, ensuring that they could make informed decisions. Then, the four agricultural green production technologies (including soil testing formula, green prevention and control, water-saving irrigation, and straw returning) with regional applicability in Shanghai were introduced to the new agricultural business entities under investigation. Finally, the team inquired about each new agricultural business entity's personal situation as well as his or her willingness to use environmentally friendly production methods and reduce pesticide and fertilizer use. A total of 109 questionnaires were distributed, with 106 valid questionnaires recovered, for a 97.2 percentile recovery rate, among which are nine large grain farmers; 20 family farms; 81 cooperatives; and 21 leading enterprises. (In China, a new agricultural business entity can operate on a variety of scales.) The types of new agricultural business entities under investigation are shown in Figure 2.

### 4.2. Statistical Analysis

SPSS version 26.0 was used to test the data for reliability and validity, and Stata version 15 was used for regression analysis and correlation tests. In this paper, regression analysis on the questionnaires is performed using the Ordered Logit Model and the Ordered Probit Model. The Logit Model follows the logical distribution, while the Probit Model follows the normal distribution; both belong to the discrete selection Model. Both models can be used to investigate ordered variables, but the Ordered Logit Model is simpler and more efficient. Therefore, the survey data was empirically analyzed with the Ordered Logit Model and robustly tested with the Ordered Probit Model.

#### 4.2.1. Ordered Logit Model

The variable *Y* is explained as “willingness of green production,” and the score range is 1 to 5. *Y* is a multivalued ordered variable. Referring to other researchers, this paper investigated decision-making willingness using the Ordered Logit Model [33]. Model 1: regression based on economic and ecological benefit perceptions, guidance, incentive, and restraint regulations, and control variables. Environmental regulation variables are obtained in Model 2 by weighting the regression coefficient ratios of guidance, incentive, and restraint regulations in Model 1. Model 2: regression based on economic and ecological benefit perceptions, environmental regulation, and control variables. The expressions of Models 1-2 are as follows:

(1) $$\begin{array}{c} \frac{P\left(Y_{i}\leq j\;|\;X\right)}{P\left(Y_{i}>j\;|\;X\right)}=\frac{P\left(Y_{i}\leq j\;|\;X\right)}{1-P\left(Y_{i}\leq j\;|\;X\right)},\;j=1,2,3,4,5. \end{array}$$

Considering Ordered Logit function,

(2) $$\begin{array}{c} \log\text{it}\left(P\left(Y_{i}\leq j\;|\;X\right)\right)=\ln\left(\frac{P\left(Y_{i}\leq j\;|\;X\right)}{P\left(Y_{i}>j\;|\;X\right)}\right)=\ln\left(\frac{P\left(Y_{i}\leq j\;|\;X\right)}{1-P\left(Y_{i}\leq j\;|\;X\right)}\right),\;j=1,2,3,4,5. \end{array}$$

The Ordered Logit is defined as

(3) $$\begin{array}{c} \ln\left(\frac{P\left(Y_{i}\leq j\;|\;X\right)}{1-P\left(Y_{i}\leq j\;|\;X\right)}\right)=-\alpha_{i}+\sum \beta_{i}X_{i}+\varepsilon ,\;j=1,2,3,4,5. \end{array}$$

Here, *Y*_*i*_ denotes the i-th new agricultural business entity's green production willingness; j denotes the willingness level; *α*_i_ denotes the intercept; *β*_*i*_ denotes the coefficient of the corresponding explanatory variable *X*_*i*_; *X*_*i*_ denotes the *i*-th explanation that affects the green production willingness variable; and *ε* denotes the random error term.

Model 3 expands on Model 2 by including a decentralized environmental regulation and economic benefit perception synergy item, as well as a decentralized environmental regulation and ecological benefit perception synergy item. Model 3: regression based on economic and ecological benefit perceptions, environmental regulation, synergy item between environmental regulation and economic benefit perception, synergy item between environmental regulation and ecological benefit perception, and control variables. The expression of Model 3 is as follows:

(4) $$\begin{array}{c} \ln\left(\frac{P\left(Y_{i}\leq j\;|\;X\right)}{1-P\left(Y_{i}\leq j\;|\;X\right)}\right)=-\alpha_{i}+\sum \beta_{i}X_{i}+\eta_{1}\left(X_{1}-{\bar{X}}_{1}\right)\left(X_{1}-{\bar{X}}_{3}\right)+\eta_{2}\left(X_{2}-{\bar{X}}_{2}\right)\left(X_{1}-{\bar{X}}_{3}\right)+\varepsilon ,\;j=1,2,3,4,5. \end{array}$$

Here, *η*_1_ denotes the coefficient of economic benefit perception and environmental regulation synergy after decentralization; *η*_2_ denotes the coefficient of ecological benefit perception and environmental regulation synergy after decentralization; *X*_1_ represents the economic benefit perception; *X*_2_ represents the ecological benefit perception; *X*_3_ represents the environmental regulation; other relevant variables are the same as Models 1-2.

#### 4.2.2. Ordered Probit Model

In this paper, the Ordered Probit Model is used to perform a robust test on Ordered Logit Models 1–3, and the maximum likelihood estimation method is used to regression the equation. The expression of Models 1-2 is as follows:

(5) $$\begin{array}{c} {\text{AGPW}}_{j}^{*}=\sum \beta_{j}X_{j}+\varepsilon_{j}. \end{array}$$

The expression of Model 3 is as follows:

(6) $$\begin{array}{c} {\text{AGPW}}_{j}^{*}=\sum \beta_{j}X_{j}+\eta_{1}\left(X_{1}-{\bar{X}}_{1}\right)\left(X_{3}-{\bar{X}}_{3}\right)+\eta_{2}\left(X_{2}-{\bar{X}}_{2}\right)\left(X_{3}-{\bar{X}}_{3}\right)+\varepsilon_{j}. \end{array}$$

AGPW_*j*_^*∗*^ is assumed to be a continuous recessive variable with *r*_*1*_, *r*_*2*_, *r*_*3*_, and *r*_*4*_ cut points. When AGPW_*j*_^*∗*^ < *r*_*1*_, the willingness of new agricultural business entities to adopt green production is very low; when *r*_*1*_ ≤ AGPW_*j*_^*∗*^ < *r*_*2*_, the willingness of new agricultural business entities to adopt green production is low; …; when *r*_*4*_ ≤ AGPW_*j*_^*∗*^, the willingness of new agricultural business entities to adopt green production is very high. Although the value of AGPW_*j*_^*∗*^ cannot be determined, the selection result of AGPW_*j*_ in response to the green production willingness of the new agricultural business entities can be obtained. When the AGPW_*j*_ selection result is between 1 and 5, it means the following:

(7) $$\begin{array}{c} {\text{AGPW}}_{j}=\left\{\begin{array}{cc} 1, & {\text{AGPW}}_{j}^{*}\leq r_{1},\\ 2, & {\text{r}}_{1}<{\text{AGPW}}_{j}^{*}\leq r_{2},\\ 3, & {\text{r}}_{2}<{\text{AGPW}}_{j}^{*}\leq r_{3},\\ 4, & {\text{r}}_{3}<{\text{AGPW}}_{j}^{*}\leq r_{4},\\ 5, & {\text{r}}_{4}<{\text{AGPW}}_{j}^{*}. \end{array}\right) \end{array}$$

Here, AGPW_j_ denotes the willingness of new agricultural management entities to produce green; *r*_1_, *r*_2_, *r*_3_, *r*_4_, *r*_5_ denote the threshold, satisfying *r*_1_ < *r*_2_ < *r*_3_ < *r*_4_ < *r*_5_; other relevant variables are the same as those of the Ordered Logit Models 1–3.

### 4.3. Variables Description

The definition and description statistics of variables are shown in Table 1.

#### 4.3.1. Explained Variable

“Agricultural green production willingness” refers to the willingness of new agricultural business entities to produce in a green manner during the agricultural production process. The explanatory variables are defined as 1–5, and the willingness to green production increases in turn.

#### 4.3.2. Core Variables

Refer to C Y Yang et al.'s and Y Z Huang et al.'s studies on economic and ecological benefit perceptions [7, 34]. The average value of “the effect of green production on agricultural product output” and “the effect of green production on agricultural product prices” is used to assess how new agricultural business entities perceive the economic benefit of green production. The average value of “the improvement effect of green production on the rural ecological environment” and “the promotion effect of green production on the sustainable development of agriculture” was chosen as the perception index of new agricultural business entities on the ecological benefit of green production. Refer to X Y Zhao et al.'s and H L Zhang et al.'s studies on environmental regulation [8, 23]. The three questions chosen to assess the government's guidance, incentive, and restraint regulations of agricultural green production are “the government's guidance intensity for agricultural green production,” “the government's incentive intensity for agricultural green production,” and “the government's punishment intensity for nongreen production.”

#### 4.3.3. Control Variables

Referring to other scholars' research [35–37], choose “age,” “number of annual agricultural training,” “agricultural income to household income ratio,” “cultivated land area,” “frequency of communication with neighbors about agricultural green production,” “green production risk,” and “green production behavior of other people in the village” as control variables. Based on the differences between the four business types of new agricultural business entities, this paper introduces a new control variable “business scale.”

## 5. Empirical Analysis

### 5.1. Model Check

Models 1–3 were tested for reliability and validity using SPSS 23. Models 1–3 have Cronbach's *α* of 0.728, 0.669, and 0.647, respectively, and reliability is greater than 0.6. Models 1–3 have KMO of 0.729, 0.722, and 0.636, respectively, and validity is greater than 0.6. Models 1–3 were found to be reliable and valid. STATA 15 was used to test Models 1–3 for collinearity. Models 1–3 have no multicollinearity issues because all VIF values are less than 4 (much less than 10). Finally, Models 1–3 can be estimated using the Ordered Logit Model.

### 5.2. Ordered Logit Regression Results for Models 1–3

The Ordered Logit Models 1–3 results are shown in Table 2 and Figure 3.

#### 5.2.1. The Direct Impact of the Perceptions of Economic Benefit and Ecological Benefit on the Willingness of New Agricultural Business Entities to Engage in Green Production

The regression results of Models 1–3 show that the perception of economic benefit has a positive impact on the willingness of new agricultural business entities to green production at significance levels of 1%, 1%, and 5%. Hypothesis H1a is verified, and the self-interested view under the Economic and Social Man Hypothesis is confirmed. The regression results of Models 1–3 show that the perception of ecological benefit has a positive impact on the willingness of new agricultural business entities to produce green at significance levels of 10%, 10%, and 5%. Hypothesis H1b is verified, and the altruistic view under the Economic and Social Man Hypothesis is confirmed. Furthermore, in Models 1–3, the economic benefit perception has a greater impact coefficient on the willingness of new agricultural business entities to engage in green production than ecological benefit perception, confirming the judgment of socialist market economic activities with Chinese characteristics in the Hypothesis of Economic and Social Man—with altruism as the guide and adjustment dominated by self-interest.

#### 5.2.2. The Direct Impact of Environmental Regulation on the Willingness of New Agricultural Business Entities to Green Production

According to the regression results of Model 1, the guidance regulation has a positive impact on the green production willingness of new agricultural business entities, but it is not significant. The H2a hypothesis has not been verified. The lack of significance of guidance regulation in Model 1 could be attributed to the close relationship between ecological benefit perception and guiding regulation, which influences the significance of guidance regulation. Therefore, the impact of guidance regulation needs to be verified by the Model with the addition of synergies. The impact of incentive regulation on the willingness of new agricultural business entities to engage in green production is minor and insignificant. The H2b hypothesis has yet to be proven. The following factors could be at play: the total amount of agricultural green production subsidies is small; the threshold for receiving agricultural green production subsidies is low; and the input cost of new agricultural business entities to green production is high. Restraint regulation has a positive impact on the willingness of new agricultural business entities to engage in green production at the 5% significance level. The H2c hypothesis has been proven. According to the regression results of Models 2-3, environmental regulation has a positive effect on the green production willingness of new agricultural business entities at the 1% and 5% significance levels. The H2 hypothesis has been proven.

#### 5.2.3. The Effect of Synergy between Benefit Perception and Environmental Regulation on the Willingness of New Agricultural Business Entities to Produce Green

According to the regression results of Model 3, the synergy item of economic benefit perception and environmental regulation has a negative impact on the green production willingness of new agricultural business entities, but it is not significant. The H3a hypothesis remains unproven. The reason for this is that as China's “green agricultural products” market has grown, the synergy effect of economic benefit perception and environmental regulation on the willingness of new agricultural business entities to produce green has weakened. The synergy item of ecological benefit perception and environmental regulation positively affects the green production willingness of new agricultural business entities at the 10% significance level. The H3b hypothesis has been proven.

#### 5.2.4. The Impact of Control Variables on the Willingness of New Agricultural Business Entities to Adopt Green Production

According to the regression results of Models 1–3, the business scale has a positive impact on the green production willingness of new agricultural business entities at significance levels of 5%, 5%, and 10%. In other words, the higher the level of business scale is, the more eager the new agricultural business entities are to produce green.

### 5.3. Robustness Check

Ordered Probit Models 1–3 were used to test the robustness of Ordered Logit Models 1–3. Except for the ecological benefit perception in the Ordered Probit Models 1–2, whose direction is consistent with the Ordered Logit Models 1–2 but not significant, the other core variables' directions and significance are consistent. It is possible that the lack of significance of ecological benefit perception in Ordered Probit Models 1-2 is due to a synergy between ecological benefit perception and environmental regulation, which affects its significance in Ordered Probit Models 1-2. Both the Ordered Probit Model without environmental regulation and the Ordered Probit Model with covariables have significant regression results for ecological benefit perception, supporting this viewpoint. Therefore, the study's findings are fairly solid. The Ordered Probit Models 1–3 regression results are shown in Table 3 and Figure 4. (The control variables are the same as those in Table 2.)

### 5.4. Extended Analysis

In order to confirm the impact of guidance regulation on new agricultural business entities' green production intentions, as well as to further investigate the synergistic effect of various regulatory means and benefit perceptions, Models 4–6 are designed to introduce the synergy between various regulatory measures and two types of benefit perception. Cronbach's coefficients are 0.625, 0.622, and 0.646 for Models 4–6, respectively. The KMOs for Models 4–6 are 0.646, 0.626, and 0.628. All VIF values are less than 4. Therefore, Models 4–6 can be estimated using the Ordered Logit Model. The regression results for Models 4–6 are shown in Table 4 and Figure 5. (The control variables are the same as in Table 2).

The perceptions of economic and ecological benefit are still significant in the regression results of Models 4–6. The H1a and H1b hypotheses have been confirmed yet again. The results of Model 4 regression show that, at a 10% level of significance, guidance regulation has a positive impact on the willingness of new agricultural business entities to engage in green production, proving hypothesis H2a; and the synergistic item of guidance regulation and ecological benefit perception positively affect the green production willingness of new agricultural business entities at a significance level of 10%. The results of Model 6 regression show that the restraint regulation positively affects new agricultural business entities' willingness to engage in green production at a 5% significance level, proving hypothesis H2c; at a significance level of 10%, the synergistic item of restraint regulation and ecological benefit perception positively affect the green production willingness of new agricultural business entities.

## 6. Conclusion and Suggestion

The primary goal of this study is to determine how benefit perception and environmental regulation affect new agricultural business entities' willingness to produce green in China. The following was discovered: first, both economic benefit perception and ecological benefit perception have a significant role in promoting the willingness of new agricultural business entities to green production, and the driving effect of economic benefit perception is stronger than ecological benefit perception. The findings verify the “Economic and Social Man Hypothesis” that people are self-interested and altruistic, as well as the Hypothesis's judgment on the behavior of “economic and social man” in the socialist market economy with Chinese characteristics. Second, environmental regulation can increase the willingness of new agricultural businesses to engage in green production. However, among the three regulatory measures, only the guidance and restraint regulations have a significant impact. Therefore, in environmental regulation, there is a phenomenon known as “relative system failure.” Third, the synergy between ecological benefit perception and environmental regulation is also the key to influencing the willingness of new agricultural business entities to green production. The extended analysis finds that the impact of ecological benefit perception on new agricultural business entities' green production willingness is dependent to some extent on guidance and restraint regulations and that the impact of guidance and restraint regulations on new agricultural business entities' green production willingness is also influenced by ecological benefit perception. Fourth, the scale of business has a great influence on the green production willingness of new agricultural business entities. It means that the higher the level of business scale is, the more eager the new agricultural business entities are to produce green products.

Based on the preceding conclusions, the following recommendations are made: first, strengthen the perceptions of the economic and ecological benefit of new agricultural business entities to green production. Measures should be taken to improve the market for green agricultural products and encourage the development of environmental protection technology for increasing production in order to improve the economic benefits of green production and strengthen the perception of economic benefits. Measures such as regularly publicizing the improvement of the agroecological environment, testing, and feedback on the soil quality of planting areas should be taken to improve the perception of ecological benefit. Second, strengthen guidance and restraint regulations and adjust incentive regulation methods. Try to change the way agricultural green production subsidies are distributed—from a one-time direct subsidy to a series of standard-compliant subsidies while also increasing spiritual incentives for agricultural green production. Third, improve the connection between ecological benefit perception and guidance regulation, as well as the connection between ecological benefit perception and restraint regulation. The propaganda of agricultural green production in guidance regulation and the education of agricultural nongreen production in restraint regulation should be aimed at improving the perception of the ecological benefits of new agricultural business entities. Fourth, cultivate the new agricultural business entities with larger business scales. Application conditions should be relaxed, and policy support should be increased, to increase the proportion of cooperatives and leading enterprises in the new agricultural business entities.

## Figures and Tables

**Figure 1:** The synergy roadmap of benefit perception and environmental regulation.

**Figure 2:** The types of new agricultural business entities under investigation.

**Figure 3:** Results of the Ordered Logit Regression Models 1–3. Notes: EEP1 means economic benefit perception, EEP2 means ecological benefit perception, ER means environmental regulation, GR means guidance regulation, IR means incentive regulation, RR means restraint regulation, EBP1 × ER means the synergy between economic benefit perception and environmental regulation, EBP2 × ER means the synergy between ecological benefit perception and environmental regulation.

**Figure 4:** Results of the Ordered Probit Regression Models 1–3. Notes: The EBP1, EBP2, ER, GR, IR, RR, EBP1 × ER, and EBP2 × ER are the same as those in Figure 3.

**Figure 5:** Results of Ordered Logit Regression Models 4–6. Notes: GR × EBP1 means the synergy between guidance regulation and economic benefit perception; GR × EBP2 means the synergy between guidance regulation and ecological benefit perception; IR × EBP1 means the synergy between incentive regulation and economic benefit perception; IR × EBP2 means the synergy between incentive regulation and ecological benefit perception; RR × EBP1 means the synergy between restraint regulation and economic benefit perception; RR × EBP2 means the synergy between restraint regulation and ecological benefit perception. The EBP1, EBP2, GR, IR, and RR are the same as those in Figure 3.

**Table 1:** Definition and description statistics of variables.

Variable	Connotation and assignment	Mean	Standard deviation
Green production willingness	Very low = 1; Low = 2; Normal = 3; High = 4; very high = 5	4	0.088
Economic benefit perception = (A1 + A2)/2	A1 very low = 1; Low = 2; Normal = 3; High = 4; very high = 5	3.80	0.079
	A2 very low = 1; Low = 2; Normal = 3; High = 4; very high = 5		
Ecological benefit perception = (B1 + B2)/2	B1 very low = 1; Low = 2; Normal = 3; High = 4; very high = 5	3.95	0.080
	B2 very low = 1; Low = 2; Normal = 3; High = 4; very high = 5		
Guidance regulation	Very low = 1; Low = 2; Normal = 3; High = 4; very high = 5	3.79	0.093
Incentive regulation	Very low = 1; Low = 2; Normal = 3; High = 4; very high = 5	3.42	0.098
Restraint regulation	Very low = 1; Low = 2; Normal = 3; High = 4; very high = 5	3.55	0.110
Age	Under 30 years old = 1; 30–40 years old = 2; 40–50 years old = 3; 50–60 years old = 4; over 60 years old = 5	2.75	0.092
Business scale	Large grain grower = 1; family farm = 2; professional cooperative = 3; big enterprise = 4	3.08	0.060
Training times per year	Did not participate = 1; 1–2 times = 2; 3–5 times = 3; 6–10 times = 4; 10 times or more = 5	2.95	0.839
Proportion of agricultural income	Below 10% = 1; 10%–40% = 2; 40%–60% = 3; 60–90% = 4; above 90% = 5	3.18	0.816
Cultivated area	0–6.67 hectares = 1; 6.67–20 hectares = 2; 20–33.33 hectares = 3; 33.33–66.67 hectares = 4; over 66.67 hectares = 5	2.62	0.839
Communication with neighbors about green production	No communication = 1; less communication = 2; Normal = 3; more communication = 4; frequent communication = 5	3.41	0.816
Green production risk	Very low = 1; Low = 2; Normal = 3; High = 4; very high = 5	2.99	0.821
Green production behavior of others	Very poor = 1; Poor = 2; Fair = 3; Good = 4; very good = 5	2.46	0.125

**Table 2:** Results of ordered logit regression models 1–3.

Variable	Model (1)	Model (2)	Model (3)
Economic benefit perception	1.014^*∗∗∗*^ (0.371)	1.012^*∗∗∗*^ (0.357)	0.954^*∗∗*^ (0.375)
Ecological benefit perception	0.623^*∗*^ (0.372)	0.623^*∗*^ (0.370)	0.792^*∗∗*^ (0.387)
Environmental regulation		1.003^*∗∗∗*^ (0.353)	0.885^*∗∗*^ (0.371)
Guidance regulation	0.429 (0.352)		
Incentive regulation	0.068 (0.292)		
Restraint regulation	0.465^*∗∗*^ (0.232)		
Economic benefit perception × environmental regulation			−0.700 (0.500)
Ecological benefit perception × environmental regulation			1.105^*∗*^ (0.567)
Age	−0.250 (0.230)	−0.251 (0.221)	−0.292 (0.223)
Business entity scale	0.712^*∗∗*^ (0.346)	0.712^*∗∗*^ (0.345)	0.634^*∗*^ (0.358)
Training times per year	−0.124 (0.201)	−0.124 (0.201)	−0.188 (0.206)
Proportion of agricultural income	0.062 (0.165)	0.062 (0.165)	0.094 (0.167)
Cultivated area	−0.107 (0.181)	−0.107 (0.178)	−0.131 (0.183)
Communication with neighbors	−0.130 (0.233)	−0.130 (0.230)	−0.190 (0.237)
Green production risks	−0.207 (0.242)	−0.207 (0.242)	−0.165 (0.249)
Production behavior of others	−0.078 (0.196)	−0.077 (0.191)	−0.073 (0.198)
Pseudo R2	0.2310	0.2310	0.2457
LR chi2 (13)	60.27^*∗∗∗*^	60.27^*∗∗∗*^	64.09^*∗∗∗*^

Notes: ^*∗∗∗*^, ^*∗∗*^, and ^*∗*^ indicate significant at a level of 1%, 5%, and 10%, respectively. The coefficients are outside the parentheses, and the robust standard errors are inside the parentheses.

**Table 3:** Regression results of Ordered Probit Models 1–3.

Variable	Model (1)	Model (2)	Model (3)
Economic benefit perception	0.603^*∗∗∗*^ (0.210)	0.603^*∗∗∗*^ (0.203)	0.559^*∗∗∗*^ (0.214)
Ecological benefit perception	0.233 (0.198)	0.233 (0.197)	0.394^*∗*^ (0.215)
Environmental regulation		0.500^*∗∗∗*^ (0.173)	0.541^*∗∗∗*^ (0.177)
Guidance regulation	0.139 (0.176)		
Incentive regulation	0.098 (0.162)		
Restraint regulation	0.263^*∗∗*^ (0.129)		
Economic benefit perception × environmental regulation			−0.353 (0.251)
Ecological benefit perception × environmental regulation			0.571^*∗∗*^ (0.261)
Control variable	Control	Control	Control
Pseudo R2	0.2242	0.2242	0.2463
LR chi2 (13)	58.48^*∗∗∗*^	58.48^*∗∗∗*^	64.26^*∗∗∗*^

**Table 4:** Regression results of Ordered Logit Models 4–6.

Variable	Model (4)	Model (5)	Model (6)
Economic benefit perception	0.935^*∗∗*^ (0.392)	0.976^*∗∗∗*^ (0.371)	1.220^*∗∗∗*^ (0.357)
Ecological benefit perception	0.940^*∗∗*^ (0.380)	0.945^*∗∗∗*^ (0.356)	0.691^*∗*^ (0.360)
Guidance regulation	0.536^*∗*^ (0.295)		
Guidance regulation × economic			
Benefit perception	−0.176 (0.368)		
Guidance regulation × ecological			
Benefit perception	0.667^*∗*^ (0.393)		
Incentive regulation		0.266 (0.256)	
Incentive regulation × economic			
Benefit perception		−0.261 (0.343)	
Incentive regulation × ecological			
Benefit perception		0.522 (0.420)	
Restraint regulation			0.485^*∗∗*^ (0.234)
Restraint regulation × economic			
Benefit perception			−0.439 (0.298)
Restraint regulation × ecological			
Benefit perception			0.628^*∗*^ (0.381)
Control variable	Controlled	Controlled	Controlled
Pseudo R2	0.2290	0.2132	0.2318
LR chi2 (13)	59.74^*∗∗∗*^	55.61^*∗∗∗*^	60.47^*∗∗∗*^

## Data Availability

All research data were obtained from in-depth interviews and questionnaires. All data included in this study are available upon request by contact with the corresponding author.
